# The Clinical Application Value of the Prognostic Nutritional Index for the Overall Survival Prognosis of Patients with Esophageal Cancer: A Robust Real-World Observational Study in China

**DOI:** 10.1155/2022/3889588

**Published:** 2022-07-13

**Authors:** Juanjuan Kang, Guishu Yang, Dongsheng Wang, Ying Lin, Qifeng Wang, Huaichao Luo

**Affiliations:** ^1^Affiliated Foshan Maternity & Child Healthcare Hospital, Southern Medical University (Foshan Maternity & Child Healthcare Hospital), Foshan 528000, China; ^2^Department of Clinical Laboratory, Sichuan Cancer Hospital & Institute, Sichuan Cancer Center, School of Medicine, University of Electronic Science and Technology of China, Chengdu 610041, China; ^3^Department of Clinical Laboratory, Guangyuan Central Hospital, Guangyuan 628099, China; ^4^Department of Laboratory Medicine, Sichuan Provincial People's Hospital, University of Electronic Science and Technology of China, Chengdu 610072, China; ^5^Department of Radiation Oncology, Sichuan Cancer Hospital & Institute, Sichuan Cancer Center, School of Medicine, University of Electronic Science and Technology of China, Chengdu 610041, China

## Abstract

Esophageal cancer is a kind of cancer with high morbidity and mortality, which is accompanied by a profound poor prognosis. A prognostic nutritional index, based on serum albumin levels and peripheral lymphocyte count, has been confirmed to be significantly associated with various cancers. This study was aimed at exploring the prognostic significance of PNI in the overall survival prognosis of patients with esophageal cancer. As a real-world study based on the big database, clinical data of 2661 patients with esophageal cancer were evaluated retrospectively, and the individuals were randomly divided into training and testing cohorts. In these two cohorts, patients are classified into a high-risk group (PNI < 49) and a low-risk group (PNI ≥ 49). Univariate and multivariate analyses were performed to analyze the independent risk factors for the prognosis of esophageal cancer patients by using the Cox proportional hazards regression model. In this study, whether in the training cohort or the testing cohort, according to the univariate analysis, gender, tumor size, tumor grade, T stage, N stage, M stage, TNM stage, and PNI were significantly correlated with overall survival. Furthermore, the multivariate analysis showed that gender, T stage, N stage, M stage, TNM stage, and PNI were independent prognostic risk factors for esophageal cancer. PNI can be regarded as an independent prognostic factor combined with gender, T stage, N stage, M stage, and TNM stage, and it might be a novel reliable biomarker for esophageal cancer.

## 1. Introduction

Esophageal cancer (EC), including the 2 most common histologic subtypes: adenocarcinoma (AC) and squamous cell carcinoma (SCC), ranks seventh in terms of incidence and sixth in mortality overall [1]. Recently, with the improvement of treatment technology and equipment and the emergence of the era of precision radiotherapy, the efficacy of esophageal cancer treatment has been improved to a certain extent, but the overall survival rate has not been significantly improved [2]. This is mainly because patients are usually at a middle and advanced stage at the time of diagnosis, which is often accompanied by lymph node or distant metastasis. Even if they were treated at this time, the prognosis of patients remains poor. In addition, it has been reported that inflammatory and nutritional status has a strong impact on the outcome of cancer treatment [3, 4]. The prognostic nutritional index (PNI) calculated by lymphocyte count and serum albumin level was originally proposed as a predictor of postoperative complications and operative morbidity of patients with gastrointestinal neoplasms, which reflects the condition of nutrition and immunity in cancer patients [5, 6]. And accumulating evidence suggests that PNI is associated with the prognosis of several cancer types, such as gastric cancer [7], lung cancer [8], breast cancer [9], and colorectal cancer [5]. To the best of our knowledge, there were a few studies suggesting that PNI is related to the prognosis of esophageal cancer. However, compared with other studies, this is the first real-world study aimed at exploring the prognostic significance of preoperative PNI in esophageal cancer patients based on such big data, and the validity of the data has been confirmed by the training and testing cohort. Real-time detection of PNI helps to improve the patients' immunity and nutritional status timely before treatment, so that the prognosis and survival of the patient can be improved.

## 2. Materials and Methods

### 2.1. Study Population

Clinical data of 2661 newly diagnosed patients with esophageal cancer who were admitted to Sichuan Cancer Hospital from January 2009 to December 2017 were collected and analyzed retrospectively. The inclusion criteria were as follows: (1) all patients who have been pathologically diagnosed with esophageal cancer and met the eighth edition of TNM staging of esophageal cancer, (2) all patients who had complete clinical data and were followed up for at least five years, and (3) complete clinical and follow-up data. The exclusion criteria were as follows: (a) any adjuvant treatment was performed before surgery, (2) any anti-inflammatory drugs were used, and (3) patients had multiple tumors. According to the above inclusion and exclusion criteria, 2661 newly diagnosed esophageal cancer patients were eventually enrolled in the study. Among them, 2173 cases were male, accounting for 81.66%, and 488 cases were female, accounting for 18.34%.

### 2.2. Data Collection

Collect the general clinical data of patients, mainly including age, gender, postoperative adjuvant treatment, Karnofsky Performance Status (KPS score), tumor size, tumor grade, tumor location, T stage, N stage, M stage, TNM stage, and PNI. Pathological TNM stages were uniformly adjusted according to the 8th edition of TNM classification, which was approved by the Union for International Cancer Control (UICC) and American Joint Committee on Cancer (AJCC) staging system in 2017. And the tumor grade was assessed based on the 1973 World Health Organization (WHO) classification guidelines [10]. The tumor size was defined as the longest diameter of the general postoperative pathological specimens. The PNI was calculated according to the formula as follows: PNI = serum albumin level (g/L) + 5∗peripheral lymphocyte count (∗10^9^/L) [6]. All patients were followed up regularly after surgery, with routine blood and biochemical tests. This study was approved by the Institutional Review Board of Sichuan Cancer Hospital & Institute.

### 2.3. Determine the Subjects of the Training Cohort and the Testing Cohort

According to the exclusion and inclusion criteria, a total of 2661 patients were evaluated in this study, and the 2661 individuals were randomly divided into training and testing cohorts. There was no overlap in the samples between the two groups. Finally, the training cohort contained 1332 subjects, and the testing cohort contained 1329 subjects.

### 2.4. Statistical Analysis

The data were analyzed with the statistical programming language R (R Foundation for Statistical Computing, https://www.r-project.org/) and IBM SPSS Statistics version 20.0 software (IBM Corp., Armonk, NY, USA). The ggplot2 package was applied in drawing the LOESS curve to choose the cutoff value of PNI [11]. The associations of clinical characteristics with PNI were evaluated by using the tableone package, using the *χ*^2^ test by default. Survival curves of overall survival (OS) were generated by the Kaplan–Meier method, while the survminer and survival packages were utilized for data visualization. Factors significant on univariate analysis were included in Cox proportional hazards multivariate models, estimating hazard ratios (HR), and 95% confidence interval (CI). All *p* values < 0.05 were considered statistically significant.

## 3. Results

### 3.1. Choosing the Cutoff Value of PNI

A LOESS smoothing curve plotting the probability of death with PNI and cut point for PNI were chosen, and the base reference corresponds to the range with the lowest mortality risk [12]. We determined the PNI value corresponding to the maximum slope cut point through the algorithm, which was used as the cutoff value to divide the research objects into a high-risk group and low-risk group. And this value is 49 as shown in Figure 1. Overall survival (OS) was defined as the time from the date of diagnosis to death or last follow-up.

### 3.2. Clinicopathological Characteristics of Patients in the Training Cohort

Of the total, there were 1332 subjects in the training cohort, the median age of the study cohort was 62 years (range: 34-90), and 1088 (81.7%) were male and 244 (18.3%) were female. According to the best cutoff value of PNI, individuals were divided into the high-risk group (PNI < 49) and low-risk group (PNI ≥ 49). There were 490 subjects in the high-risk group and 842 subjects in the low-risk group. No significant differences were noted in the KPS score, tumor grade, tumor location, T stage, N stage, M stage, and TNM stage between the two groups, while comparing the age (*p* < 0.001), postoperative adjuvant treatment (*p* = 0.003), gender (*p* < 0.001), and tumor size (*p* < 0.001) of the two groups, the differences are statistically significant in the high-risk group and low-risk group (Table 1).

### 3.3. Survival Analysis of the PNI Group in the Training Cohort

The median patient follow-up time was 27.4 months. The OS rate was significantly worse in the high-risk group compared with the low-risk group (*p* = 0.0075) (Figure 2). The one-, three-, and five-year OS rate was 83.4%, 53.4%, and 39.7% in the high-risk group, respectively, while the one-, three-, and five-year OS rate was 88%, 57.2%, and 43.6%, respectively, in the low-risk group (Figure 2).

### 3.4. Prognostic Factors of Overall Survival in the Training Cohort

To confirm the significance of PNI in overall survival, univariate and multivariate analyses were performed. The univariate and multivariate analyses of clinicopathological factors for OS are shown in Table 2. According to the univariate analysis, gender (HR = 0.623, 95% CI: 0.501-0.775, *p* < 0.001), tumor size (HR = 0.754, 95% CI: 0.643-0.883, *p* < 0.001), tumor grade (*p* < 0.05), T stage (HR = 0.687, 95% CI: 0.624-0.757, *p* < 0.001), N stage (HR = 0.591, 95% CI: 0.546-0.639, *p* < 0.001), TNM stage (HR = 0.566, 95% CI: 0.519-0.618, *p* < 0.001), and PNI (HR = 1.114, 95% CI: 1.029-1.206, *p* = 0.008) were significantly correlated with OS. Furthermore, the multivariate analysis showed that gender (HR = 0.702, 95% CI: 0.563-0.875, *p* = 0.002), T stage (HR = 0.639, 95% CI: 0.524-0.779, *p* < 0.001), N stage (HR = 0.553, 95% CI: 0.461-0.663, *p* < 0.001), TNM stage (HR = 0.480, 95% CI: 0.390-0.591, *p* < 0.001), and PNI (HR = 1.186, 95% CI: 1.012-1.391, *p* = 0.036) were independent prognostic risk factors.

### 3.5. Clinicopathological Characteristics of Patients in the Testing Cohort

Of the total, there were 1329 subjects in the testing cohort, the median age of the study cohort was 62 years (range: 35-85), and 1085 (81.6%) were male and 244 (18.4%) were female. Patients were divided into the high-risk group and low-risk group in the testing cohort as well. There were 502 subjects in the high-risk group, while 827 subjects in the low-risk group. No significant differences were noted in the KPS score, tumor grade, tumor location, N stage, M stage, and TNM stage between the two groups, while comparing the age (*p* < 0.001), postoperative adjuvant treatment (*p* = 0.016), gender (*p* = 0.015), tumor size (*p* = 0.001), and T stage (*p* = 0.001) of the two groups, the differences are statistically significant in the two groups (*p* < 0.05) (Table 3).

### 3.6. Survival Analysis of the PNI Group in the Testing Cohort

The median patient follow-up time was 27.2 months. The OS rate was significantly worse in the high-risk group compared with the low-risk group (*p* = 0.0012) (Figure 3), which is the same as the overall survival analysis result of the training cohort. The one-year, three-year, and five-year OS rate was 82.6%, 55.7%, and 43.8% in the high-risk group separately, while the one-year, three-year, and five-year OS rate was 91.1%, 61.6%, and 49.1%, respectively, in the low-risk group.

### 3.7. Prognostic Factors of Overall Survival in the Testing Cohort

To confirm the significance of PNI in overall survival, univariate and multivariate analyses were also performed in the testing cohort. The univariate and multivariate analyses of clinicopathological factors for OS are shown in Table 4. According to the univariate analysis, gender (HR = 0.74, 95% CI: 0.655-0.836, *p* < 0.001), tumor size (HR = 0.764, 95% CI: 0.705-0.829, *p* < 0.001), tumor grade (*p* < 0.05), T stage (HR = 0.637, 95% CI: 0.574-0.706, *p* < 0.001), N stage (HR = 0.566, 95% CI: 0.521-0.615, *p* < 0.001), M stage (HR = 0.219, 95% CI: 0.133-0.361, *p* < 0.001), TNM stage (HR = 0.542, 95% CI: 0.494-0.596, *p* < 0.001), and PNI (HR = 1.145, 95% CI: 1.055-1.243, *p* = 0.001) were significantly correlated with OS. Furthermore, the multivariate analysis showed that gender (HR = 0.677, 95% CI: 0.529-0.866, *p* = 0.002), tumor size (HR = 0.8, 95% CI: 0.674-0.949, *p* = 0.01), T stage (HR = 0.601, 95% CI: 0.484-0.745, *p* < 0.001), N stage (HR = 0.584, 95% CI: 0.482-0.708, *p* < 0.001), M stage (HR = 0.12, 95% CI: 0.044-0.329, *p* < 0.001), TNM stage (HR = 0.473, 95% CI: 0.38-0.588, *p* < 0.001), and PNI (HR = 1.212, 95% CI: 1.027-1.431, *p* = 0.023) were independent prognostic risk factors (Table 4). The multivariate analysis in both training and testing cohorts showed that gender, T stage, N stage, M stage, TNM stage, and PNI were stable independent prognostic risk factors for esophageal cancer.

## 4. Discussion

In this study, whether in the training or testing cohort, our results revealed that the OS rates of the high-risk group were significantly lower than those of the low-risk group. And the univariate and multivariate analyses investigated that gender, T stage, N stage, M stage, TNM stage, and PNI were independent prognostic factors associated with OS in patients with esophageal cancer. Therefore, there were a few studies that have shown the prognostic value of PNI in esophageal cancer patients. Nakatani et al. suggested that preoperative PNI is a useful marker for predicting the long-term outcomes of EC patients undergoing NAC and subsequent subtotal esophagectomy [13]. Okadome et al. found that PNI and TIL score expression was associated with the clinical outcome in esophageal cancer, supporting their role as prognostic biomarkers [14]. Wang et al. found that the NRS2002 scores and PNI are simple and useful markers for predicting the long-term outcome in patients with esophageal cancer after CRT [15]. However, this is the first real-world observational study in China about the value of PNI for the OS prognosis of patients with esophageal cancer.

The presence of an inflammatory response is considered a pathogenic factor in the development of cancer-related malnutrition, leading to the patient's poor performance status and increased mortality after surgery [16]. Inflammatory factors are important regulators of tumor cell growth, angiogenesis, invasion, and metastasis by recruiting T lymphocytes, tumor-associated macrophages, and circulating cytokines [17, 18]. According to the calculation formula of PNI, low PNI value indicates low serum albumin level and low lymphocyte level in the patient. Low serum albumin indicates that the body is in a state of malnutrition, which is a serological indicator of the body in a state of continuous inflammation [19], while low lymphocyte level means that antitumor immune response to tumors is weakened and the imbalanced immune state in patients promotes tumor progression [20].

The univariate and multivariate results of the training cohort and the testing cohort showed that TNM stages are also independent risk factors for the prognosis of esophageal cancer; the prognosis of patients with stage III+IV is worse than that of patients with I+II, which is consistent with the research results of scholars such as RICE [21]. And T stage, N stage, and M stage are also independent risk factors for esophageal cancer. PNI is also closely related to these clinicopathological characteristics. Patients with stages III-IV have lower PNI values, and their tumor tissues are larger and often accompanied by tumor invasion and lymph node and distant metastasis, carrying a worse prognosis. And for patients with distant metastases, the risk of death is 1.591 times that for those without distant metastases, and the prognosis is very poor [22, 23]. Therefore, according to the patient's treatment willingness, reasonable palliative treatment is the main treatment method.

The results of the training cohort and the testing cohort show that the gender distribution of esophageal cancer patients in the low-risk group and high-risk group is different, and gender is also an independent risk factor for esophageal cancer, which is related to bad life and eating habits. The main clinicopathological type of esophageal cancer in China is squamous cell carcinoma. Heavy drinking and smoking are an important cause of esophageal squamous cell carcinoma, while studies have shown that the smoking rate and drinking rate of men are much higher than those of women, which has a profound impact on the effect of tumor treatment, leading to a poor prognosis [24]. In addition, Hudry et al. found that human intestinal epithelial stem cells have “gender identity” in the differentiation process [25]. In addition to obvious differences in morphology, intestinal epithelial cells of different genders have completely different responses to oncogene mutations. Is there such a difference in “gender identity” in the epithelial cells of patients with esophageal cancer? This may be another important reason for the difference in survival of patients of different genders, but it remains to be studied.

## 5. Conclusions

In conclusion, PNI can be measured at low cost, routinely and easily in clinical practice, and reflects the body's nutritional and immune status. It can be used as an index to predict postoperative survival of patients with esophageal cancer, combined with T stage, N stage, M stage, and TNM stage. For patients with low preoperative PNI values, individualized nutritional support programs should be developed to actively correct malnutrition and immune system disorders to improve the survival prognosis of patients.

## Figures and Tables

**Figure 1:** LOESS smoothing curve plotting the probability of death against PNI. The maximum slope point was used as the cutoff value.

**Figure 2:** Overall survival (OS) curve according to the PNI, based on the high-risk group (blue line) and low-risk group (red line) in the training cohort.

**Figure 3:** OS curves according to the PNI, based on the high-risk group (blue line) and low-risk group (red line) in the testing cohort.

**Table 1:** Patients' characteristics in the training cohort.

Variables	Overall (%)	PNI		*p* value
		High risk (PNI < 49)	Low risk (PNI ≥ 49)	
*n*	1332	490	842	
Age				<0.001
≤60	548 (41.1)	160 (32.7)	388 (46.1)	
>60	784 (58.9)	330 (67.3)	454 (53.9)	
Postoperative adjuvant treatment				0.003
No	720 (54.1)	291 (59.4)	429 (51.0)	
Yes	612 (45.9)	199 (40.6)	413 (49.0)	
Gender				<0.001
Female	244 (18.3)	65 (13.3)	179 (21.3)	
Male	1088 (81.7)	425 (86.7)	663 (78.7)	
KPS score				1
≥80	1327 (99.6)	488 (99.6)	839 (99.6)	
≤70	5 (0.4)	2 (0.4)	3 (0.4)	
Tumor size				<0.001
<5 cm	900 (67.6)	298 (60.8)	602 (28.5)	
≥5 cm	432 (32.4)	192 (39.2)	602 (28.5)	
Tumor grade				0.963
Well differentiated	251 (18.8)	93 (19.0)	158 (18.8)	
Moderate differentiated	521 (39.1)	195 (39.8)	326 (38.7)	
Poorly differentiated	522 (39.2)	189 (38.6)	333 (39.5)	
Other	38 (2.9)	13 (2.7)	25 (3.0)	
Tumor location				0.185
Lower chest	293 (22.0)	121 (24.7)	172 (20.4)	
Middle chest	712 (53.5)	255 (52.0)	457 (54.3)	
Upper chest	327 (24.5)	114 (23.3)	213 (25.3)	
T stage				0.295
T0-2	405 (30.4)	140 (28.6)	265 (31.5)	
T3-4	927 (69.6)	350 (71.4)	577 (68.5)	
N stage				0.865
N0-1	970 (72.8)	355 (72.4)	615 (73.0)	
N2-3	362 (27.2)	135 (27.6)	227 (27.0)	
M stage				0.784
M0	1331 (99.9)	489 (99.8)	842 (100.0)	
M1	1 (0.1)	1 (0.2)	0 (0.0)	
TNM stage				0.241
0-II	581 (43.6)	203 (41.4)	378 (44.9)	
III-IV	751 (56.4)	287 (58.6)	464 (55.1)	

**Table 2:** Univariate and multivariate Cox proportional hazards regression analyses of OS in patients of the training cohort.

Variable	Univariate		Multivariate	
	HR (95% CI)	*p* value	HR (95% CI)	*p* value
Age (60/>60)	0.944 (0.807-1.103)	0.467		
Postoperative adjuvant treatment (no/yes)	1.036 (0.888-1.208)	0.653		
Gender (female/male)	0.623 (0.501-0.775)	<0.001	0.702 (0.563-0.875)	0.002
KPS score (≥80/≤70)	0.482 (0.180-1.290)	0.146		
Tumor size (<5 cm/≥5 cm)	0.754 (0.643-0.883)	<0.001	1.009 (0.855-1.190)	0.918
Tumor grade				
Well differentiated	1 (reference)		1 (reference)	
Moderate differentiated	1.458 (1.159-1.835)	0.001	1.235 (0.979-1.559)	0.075
Poorly differentiated	1.479 (1.176-1.86)	0.001	1.165 (0.922-1.473)	0.201
Other	0.533 (0.278-1.022)	0.058	0.977 (0.505-1.890	0.945
Tumor location				
Lower chest	1 (reference)			
Middle chest	0.922 (0.758-1.121)	0.414		
Upper chest	0.984 (0.789-1.226)	0.883		
T stage (T0-2/T3-4)	0.687 (0.624-0.757)	<0.001	0.639 (0.524-0.779)	<0.001
N stage (N0-1/N2-3)	0.591 (0.546-0.639)	<0.001	0.553 (0.461-0.663)	<0.001
M stage (M0/M1)	0.572 (0.214-1.526)	0.264		
TNM stage (I-II/III-IV)	0.566 (0.519-0.618)	<0.001	0.480 (0.390-0.591)	<0.001
PNI (<49/≥49)	1.114 (1.029-1.206)	0.008	1.186 (1.012-1.391)	0.036

**Table 3:** Patients' characteristics in the testing cohort.

Variables	Overall (%)	PNI		*p* value
		High risk (PNI < 49)	Low risk (PNI ≥ 49)	
*n*	1329	502	827	
Age				0.003
≤60	546 (41.1)	180 (35.9)	366 (44.3)	
>60	783 (58.9)	322 (64.1)	461 (55.7)	
Postoperative adjuvant treatment				0.016
No	702 (52.8)	287 (57.2)	415 (50.2)	
Yes	627 (47.2)	215 (42.8)	412 (49.8)	
Gender				0.015
Female	244 (18.4)	75 (14.9)	169 (20.4)	
Male	1085 (81.6)	427 (85.1)	658 (79.6)	
KPS score				1
≥80	1324 (99.6)	500 (99.6)	824 (99.6)	
≤70	5 (0.4)	2 (0.4)	3 (0.4)	
Tumor size				0.001
<5 cm	898 (67.6)	311 (62.0)	587 (71.0)	
≥5 cm	431 (32.4)	191 (38.0)	240 (29.0)	
Tumor grade				0.953
Well differentiated	236 (17.8)	92 (18.3)	144 (17.4)	
Moderate differentiated	540 (40.6)	205 (40.8)	335 (40.5)	
Poorly differentiated	516 (38.8)	192 (38.2)	324 (39.2)	
Other	37 (2.8)	13 (2.6)	24 (2.9)	
Tumor location				0.846
Lower chest	280 (21.1)	105 (20.9)	175 (21.2)	
Middle chest	706 (53.1)	263 (52.4)	443 (53.6)	
Upper chest	343 (25.8)	134 (26.7)	209 (25.3)	
T stage				0.037
T0-2	420 (31.6)	141 (28.1)	279 (33.7)	
T3-4	909 (68.4)	361 (71.9)	548 (66.3)	
N stage				0.168
N0-1	993 (74.7)	364 (72.5)	629 (76.1)	
N2-3	336 (25.3)	138 (27.5)	198 (23.9)	
M stage				1
M0	1325 (99.7)	500 (99.6)	825 (99.8)	
M1	4 (0.3)	2 (0.4)	2 (0.2)	
TNM stage				0.132
0-II	579 (43.6)	205 (40.8)	374 (45.2)	
III-IV	750 (56.4)	297 (59.2)	453 (54.8)	

**Table 4:** Univariate and multivariate Cox proportional hazards regression analyses of OS in patients of the testing cohort.

Variable	Univariate		Multivariate	
	HR (95% CI)	*p* value	HR (95% CI)	*p* value
Age (60/>60)	0.943 (0.801-1.111)	0.483		
Postoperative adjuvant treatment (no/yes)	1.004 (0.926-1.088)	0.928		
Gender (female/male)	0.74 (0.655-0.836)	<0.001	0.677 (0.529-0.866)	0.002
KPS score (≥80/≤70)	1.136 (0.568-2.275)	0.718		
Tumor size (<5 cm/≥5 cm)	0.764 (0.705-0.829)	<0.001	0.8 (0.674-0.949)	0.01
Tumor grade				
Well differentiated	1 (reference)		1 (reference)	
Moderate differentiated	1.475 (1.153-1.886)	0.002	1.232 (0.96-1.581)	0.101
Poorly differentiated	1.565 (1.225-1.997)	<0.001	1.428 (1.114-1.831)	0.005
Other	0.314 (0.127-0.773)	0.012	0.567 (0.228-1.407)	0.221
Tumor location				
Lower chest	1 (reference)			
Middle chest	1.059 (0.857-1.310)	0.595		
Upper chest	1.129 (0.892-1.429)	0.314		
T stage (T0-2/T3-4)	0.637 (0.574-0.706)	<0.001	0.601 (0.484-0.745)	<0.001
N stage (N0-1/N2-3)	0.566 (0.521-0.615)	<0.001	0.584 (0.482-0.708)	<0.001
M stage (M0/M1)	0.219 (0.133-0.361)	<0.001	0.12 (0.044-0.329)	<0.001
TNM stage (I-II/III-IV)	0.542 (0.494-0.596)	<0.001	0.473 (0.38-0.588)	<0.001
PNI (<49/≥49)	1.145 (1.055-1.243)	0.001	1.212 (1.027-1.431)	0.023

## Data Availability

The clinical data used to support the findings of this study are available from the corresponding author upon request.
